The article "Investigations on Brain Tumor Classification Using Hybrid Machine Learning Algorithms" was published in 2022. Journal: J Healthc Eng.

# Investigations on Brain Tumor Classification Using Hybrid Machine Learning Algorithms

**DOI:** 10.1155/2022/2761847

**Published:** 2022-02-14

**Authors:** S. Rinesh, K. Maheswari, B. Arthi, P. Sherubha, A. Vijay, S. Sridhar, T. Rajendran, Yosef Asrat Waji

**Affiliations:** ^1^Department of Computer Science and Engineering, Jigjiga University, Jijiga, Ethiopia; ^2^Department of Computer Science and Engineering, CMR Technical Campus, Hyderabad, Telangana, India; ^3^Department of Computer Science and Engineering, College of Engineering and Technology, SRM Institute of Science and Technology, SRM Nagar,Kattankulathur,Kanchipuram, Chennai, Tamil Nadu, India; ^4^Department of Information Technology, Karpagam College of Engineering, Coimbatore, Tamil Nadu, India; ^5^Department of Business Administration and Information Systems, Arba Minch University, Sawla Campus, Ethiopia; ^6^Department of Computer Science and Engineering, Saveetha School of Engineering, Saveetha Institute of Medical and Technical Sciences, Chennai, Tamil Nadu, India; ^7^Makeit Technologies (Center for Industrial Research), Coimbatore, Tamil Nadu, India; ^8^Department of Chemical Engineering, College of Biological and Chemical Engineering, Addis Ababa Science and Technology University,Addis Ababa, Ethiopia

## Abstract

The imaging modalities are used to view other organs and analyze different tissues in the body. In such imaging modalities, a new and developing imaging technique is hyperspectral imaging. This multicolour representation of tissues helps us to better understand the issues compared to the previous image models. This research aims to analyze the tumor localization in the brain by performing different operations on hyperspectral images. The tumor is located using the combination of *k*-based clustering processes like *k*-nearest neighbour and *k*-means clustering. The value of *k* in both methods is determined using the optimization process called the firefly algorithm. The optimization processes reduce the manual calculation for finding *K*'s optimal value to segment the brain regions. The labelling of the areas of the brain is done using the multilayer feedforward neural network. The proposed technique produced better results than the existing methods like hybrid *k*-means clustering and parallel *k*-means clustering by having a higher peak signal-to-noise ratio and a lesser mean absolute error value. The proposed model achieved 96.47% accuracy, 96.32% sensitivity, and 98.24% specificity, which are improved compared to other techniques.

## 1. Introduction

The increasing growth of medical image analysis uses various advanced image processing techniques [1]. Due to this development, incurable diseases can be cured nowadays. This development helps to cure most life-threatening diseases like tumors, blood clots, and cancer at the initial stages. These life-threatening diseases are confirmed with the help of images of the infected region and biopsy. Mostly, the infected region's images are the first step in diagnosing the conditions [2]. The diseases are confirmed with the help of a biopsy. In such a situation, the infected regions' modeling should be highly accurate and easily visualizable.

The article "Investigations on Brain Tumor Classification Using Hybrid Machine Learning Algorithms" was published in 2022. Journal: J Healthc Eng.

This paper discusses such modeling, which is called hyperspectral imaging, to locate the abnormal growth of cells in the brain. This hyperspectral image provides an accurate result compared with other images. In general, brain activities are recorded with the help of scanning and radiogram methods. The scanning so far used for the brain is the MRI scan and CT scan [3]. MRI is the abbreviation of magnetic resonance imaging, mainly used for the body's soft tissue analysis [4]. CT is the abbreviation of computed tomography imaging used to analyze the hard tissues of the body.

MRI scanning is mainly preferred for brain analysis. The advantages of this type of scanning are the ability to view the soft tissue clearly. It does not produce any side effects because of not using any ionizing radiation to visualize the brain regions. The MRI scan is highly used to locate the abnormal growth of cells in the brain. This imaging scheme produces the brain's imaging in a greyscale format [5], which medical experts can analyze. An in-depth diagnosis is required in this imaging model to locate the tumor.

Apart from MRI scanning, other types of scanning also produce the images in a greyscale format except for the color Doppler scan. However, alternative techniques like postprocessing for segmenting the tissue regions are not producing desired results. Hence, to overcome this drawback, a new imaging technique called hyperspectral imaging is used to analyze the body's soft tissues.

Hyperspectral imaging is used in remote sensing for vegetation classification by taking pictures of hundreds of bands' regions. This imaging process is also used for capturing the brain with 128 bands. Based on the image processing techniques, the hyperspectral image is classified. These hyperspectral images represent the brain regions in different colors, which effectively understand the brain tissues. This mainly helps the doctor during the surgery process to remove the abnormal tissues. This imaging technique also helps the patient understand the current stage of their diseases due to the representation of tissues in different colors. The high-resolution camera captures the brain tumor [6].

The article "Investigations on Brain Tumor Classification Using Hybrid Machine Learning Algorithms" was published in 2022. Journal: J Healthc Eng.

This paper discussed the mapping process of the brain to locate the abnormal tissues. The technique used for the mapping was noise removal to remove any artifacts in the images for postprocessing. The segmentation process was done using a hybrid *k*-based clustering process [4]. The algorithm for optimization was utilized to choose the value of clusters for the clustering process. The neural-based labelling process was to mention the tissues of the brain in different colors. Based on the image classification accuracy, the mean absolute error value, and the peak signal-to-noise ratio, the results are compared with existing image classification methods and neural network models.

This paper is organized as follows: Section 2 discusses the various research works of tumor localization.  Section 3 presents a detailed explanation of the proposed methodologies.  Section 4 discusses the comparison of various techniques by practical implementation and evaluation.  Section 5 is about the conclusion statement based on the results and analysis.

## 2. Related Works

Hemanth et al. [1] proposed the abnormal brain image using the deep convolution method. This brain image was classified based on the dataset. The deep convolution neural network was applied to reduce design complexity. The convolution neural network model used a deep learning technique, that is, DCNN. The abnormal brain tumor dataset was used for classifying the image. Here, three layers in DCNN were carried out to perform the classification. The first layer was the convolution layer, which provides the higher-level features with trained parameters. The second layer was the ReLU Layer, which rectifies the linear unit layer. The final one was the Max-Pool layer. It was used after getting the four-cluster region. It classified the terms of metastasis, meningioma, glioma, and astrocytoma.

Deep-seated diseases like MS affect the nerve systems since they would be predicted earlier. Halimeh and Teshnehlab [2] proposed the tumors and MS simultaneous classification and diagnosis with the convolution neural network's help. Here, the image processing technique was used to classify that image, and it was diagnosed. Here, CNN was used. The MRI image was taken for the classification process of the internal image pixel's multiplications. This detects the infected area, lesion, and tumor after diagnosis.

Dong et al. [7] proposed a Farrow structure to apply the time delay filter contrary to a linear FIR structure to fulfill the requirement for real-time updates and be entirely suitable for the FPGA domain. Besides, another off-line approach was implemented to evaluate the Farrow filter coefficient if the coefficient was symmetric. Simulations have been generated to represent the structural model to the Farrow filter developed. The results likewise showed the Frost broadband adaptive antenna with a Farrow filter effectively diminishes the obstacle.

The article "Investigations on Brain Tumor Classification Using Hybrid Machine Learning Algorithms" was published in 2022. Journal: J Healthc Eng.

Choi and Jeong [8] proposed a model utilizing Speckle Reducing Anisotropic Diffusion (SRAD), guided filter, and soft thresholding to eliminate SAR image speckle noise while maintaining edge data efficiently. Initially, the generated procedure obtained a filtered image by executing an SRAD filter onto the noisy image. Thus, a logarithmic shift was used to change it to additional noise for future expulsion of the filtered image's multiplicative noise. The filtering image was transformed, using DWT, into multiresolution images. For each high and low-frequency, subimage soft thresholding and the directed filter were used. The denoised images were equipped with Inverse DWT (IDWT) and the exponential transform, showing that the procedure demonstrated superior function over the traditional filtering method and the output was both subjective and objective.

Mafi et al. [9] developed an image denoising technique within related speckle noise and Gaussian noises. The dual-tree complex wavelets transform was used on the images to accomplish a unique coefficient describing these noises. Hence, these isolated coefficients were evacuated by thresholding, and the inverse wavelet transform was executed to achieve the remake image. A connection between the dual-tree and standard wavelet-based denoising filter was applied depending on different basic parameters. Lastly, to expel some other existing noises, a spatial denoising filter was used on the image. The clinical ultrasound images are degenerated by the noise sequences. Such noise sequences helps the researchers' to understand the impacts of Gaussian and speckle noises with the help of most effective speckle and Gaussian denoising filters.

Choi and Jeong [10] proposed an algorithm utilizing SRAD and a guided filter for speckle noise decreasing and edge security. At first, speckle, which was a multiplicative noise, was detached by utilizing SRAD. The existing noise in the filtered image was transformed to added noise using algebraic transform. The additional noise that exists in the filtered image was further detached utilizing a guided filter. Lastly, the image without noise was derived utilizing aggressive transformation, indicating that the model have better noise reduction and edge-preserving capabilities than the standard filtering method.

Marie and Alalyani [11] proposed a novel firefly algorithm-based feature selection process. This also manages the Arabic text classification that was not successfully concentrated because of the Arabic language's inconvenience. This technique has been profitably tested in various complicated issues. Moreover, it has not been included in selecting feature methods to manage the classification of Arabic text. The SVM classifier was utilized as three-calculation parts for approving this method, including accuracy, recall, and F-measure. This work accomplished an accuracy of 0.994 using OSAC dataset.

The article "Investigations on Brain Tumor Classification Using Hybrid Machine Learning Algorithms" was published in 2022. Journal: J Healthc Eng.

Narayanan et al. [5] proposed a technique to access the standard EEG signal. At first, the peak EEG signal voltage estimation is computed. Finally, a developed time-frequency transformation method was used to send the signals into an image depending on the wavelet transform. Additionally, the S-transform access was planned to disengage the main features of signals to the classifier scheme. The firefly algorithm-based method was further treated to select the principal features of the signal utilized for training and testing the classifying method. In this method, the SVM, RF, and KNN methods were developed. Hence, the performance obtained an average accuracy of 80.39%. The performance affirmed that this method offered a better outcome on the chosen EEG signal.

Mashhour et al. [12] proposed a new classifier method depending on a firefly algorithm made as a managed learning algorithm. Hence, the analysis depended on the firefly algorithm created by simulating a firefly's character to bring different mates, dependent on intensity and distance. The procedure of this algorithm contained three stages. The feature selection stage was utilized to reduce the features and to select the most valuable features. The model development stage was significant in determining the firefly class moderators. The model forecast stage was utilized to apportion the testing or concealed sample in their related classes using class contributors. A few datasets ended up being related to the Ant-Miner technique. The experiment demonstrated that the firefly algorithm was the best.

Tawahid and Dsouza [13] presented an algorithm known as the Hybrid Binary Bat Enhanced Particle Swarm Optimization (HBBEPSO). In this method, a bat based genetic algorithm is used to analyze the feature space using echolocation and improved rendition of the PSO to achieve better solution in the search place. The algorithm's overall efficiency and technique were identified as the best compared to the other methods examined. Hence, the result has demonstrated the algorithm's capacity to discover the feature space for optimal feature sequence.

Sangaiah and Kumar [14] proposed an algorithm that used a relief attribute reduction with GA based on entropy for breasts cancer identification. This method's hybrid sequence was utilized to deal with the dataset with a higher dimension and concern. The information was accomplished from the WISCONSIN datasets, and the information has been classified depending on various properties. The technique was calculated and compared with the other notable feature selection processes. The experimental outcome indicates that the work has a remarkable capacity to create a decreased subspace of critical features while generating significant classifications accuracy for massive datasets.

The article "Investigations on Brain Tumor Classification Using Hybrid Machine Learning Algorithms" was published in 2022. Journal: J Healthc Eng.

Harithaa [15] presented the firefly and cuckoo search-based algorithms of feature selection with detached high accuracy and lower training upward for the PIMA Indian diabetic dataset from UCI. The empirical setup was made with the UCI dataset with the KNN classifier. The precision, accuracy, and recall were analyzed to calculate parameters, and the results were compared with those of the firefly and cuckoo search algorithms. This technique traditionally obtained high accuracy.

Long et al. [16] developed a heart disease diagnostic model with rough sets based on feature reductions and type 2 fuzzy logic (IT2FLS) intervals. Analysis among irregular groups based on feature reduction and IT2FLS targets address the issue and concern of high-dimensional datasets. IT2FLS used a hybrid teaching procedure to compose a fuzzy c-means clustering approach and the adjustment criterion by firefly chaos and hybrid genetic algorithms. This teaching procedure was costly in computational terms, especially when hired with a high-dimensional set of data. The rough set-based quality decline utilizing a chaos firefly approach was analyzed to detect an optimal reduction, reduce computational liability, and improve IT2FLS performance. Results explained remarkable device stability associated with numerous machine learning algorithms like Naive Bayes, ANN, and SVM. This model has been useful in diagnosing heart disease.

Cortes et al. [17] developed an approach for adaptively learning artificial neural networks (ADANET). It was based on analytical methods, including data-dependent generalized, which are proved in detail. The large-scale operations on the various binary division tasks are obtained using the CIFAR-10 dataset. Results explained that this technique could automatically learn network structures with very reasonable work accuracy when related to those obtained for neural networks.

Esfe et al. [18] analyzed nanofluids' thermal conductivity utilizing neural networks, test data, and correlativity for modeling thermal conductivity. Using a KD2-Pro thermal analyzer, the thermal conduction of Mg(OH)_2_ nanoparticles with a 10 nm mean diameter isolated in ethylene glycol was solved. An experimental collaboration has been developed as far as volume fraction and temperature were concerned, based on observational information at other substantial volume portions and temperature. Therefore, the relative thermal conduction as temperature and volume fraction activities was proposed through a neural network depending on the analyzed information. A system with two layers hidden in each layer and five neurons has the slightest error and a high fitting coefficient. Besides correlating the model and the correlativity obtained from test knowledge, the neural network was highly accurate and predicted the thermal conduction of Mg(OH)_2_-EG nanofluids.

The article "Investigations on Brain Tumor Classification Using Hybrid Machine Learning Algorithms" was published in 2022. Journal: J Healthc Eng.

Erkaymaz et al. [19] researched the work of two various feedforward neural networks (FFNN) for diabetes diagnosis. They used input as PIMA Indians Diabetic Dataset. The previous information indicated that the Watts–Strogatz small world FFNN delivered a good analysis work compared to traditional FFNN. Consequently, the result was associated with the Newman–Watts small world FFNN, and they demonstrated that the latter was even better. However, the Newman–Watts small world FFNN results from better output parameters were validated.

Torti et al. [20] executed an alternative analytical comprehension of the challenge from a smooth optimization perspective. Hence, the specific teaching of limited samples and acceptable conditions was analyzed using a critical point to set up any local minimal to be globally minimal. Additionally, an advanced algorithm, known as the Generalized Gauss-Newton (GGN), was returned as a surmised Newton's algorithm that moves the property of being locally united to a global minimum under the state of accurate teaching.

Hao et al. [21] proposed a glioblastoma brain tumor classification model using HSI images. The spatial and spectral features of HSI images were used by implementing various deep learning models for the detection of brain tumor. These features extracted could support obtaining accurate results in detecting brain tumor. The brain tumor detection process includes the processes like spectral phasor analysis and data oversampling, 1D-DNN-based spectral HSI feature extraction and classifications, 2D-CNN-based spectral-spatial HSI feature extraction and classifications, edge-preserving filtering-based classification results fusion and optimizations, and fully convolutional networks- (FCN-) based background segmentation.

## 3. Proposed Method

In this paper, a classification and detection model of brain tumor using hyperspectral imaging (HSI) is proposed. The brain tumor mapping technique was used in this work for improving the performance of the proposed model to achieve accurate results in terms of detecting brain tumor. The proposed model includes preprocessing, filtering, optimization, clustering, labelling, and classification processes in order to detect the brain tumor.

The article "Investigations on Brain Tumor Classification Using Hybrid Machine Learning Algorithms" was published in 2022. Journal: J Healthc Eng.

Mapping is the process, which represents the different regions of the same properties in different colors. This mapping process is used to understand the areas more effectively. This paper discusses such a mapping process for locating the abnormal tissues in the brain. The term abnormal tissue was the tumor cell whose growth was increasing without any ordered form [22, 23].

The mapping process is done on the hyperspectral image of the brain. The noise removal algorithm to remove any unwanted pixels or disturbance in the image processes the hyperspectral image. This noiseless image is suitable for a better mapping process. The mapping is carried out in two stages. The initial step is to group pixels of the same characteristics using an optimized hybrid *k*-based clustering process [24]. The second stage is to label the grouped pixels using the neural scheme.  Figure 1 is the pictorial representation of the proposed system.

### 3.1. Image Modeling

The mapping of a brain region is done using hyperspectral images. The image used in this paper is obtained from the in vivo hyperspectral format. The input image consists of 128 bands, and its color wavelength ranges from 400 to 1300 nm, that is, the bandwidth of electromagnetic radiation.

NASA usually performs mapping in hyperspectral images remote sensing application form specifying the different crops. NASA is currently performing this mapping process in the mammogram images using the MEDSEG analyzer to represent the breast region's various tissues to detect the cancer part. The migration to hyperspectral medical imaging helps to capture the images in pixels and their wide range of frequencies.

Hyperspectral imaging's main advantage is to capture the spatial and spectral information of the images through spatial and spectral scanning of the body with different wavelengths.

The information is higher due to the capture of the body of more than eight bands. Each band of the hyperspectral image holds a different story on the brain's particular region, which is impossible in the other imaging models. This paper tests the proposed hybrid firefly and *k*-based mapping in the dataset used in the parallel *k*-means clustering process. The HSI brain image is obtained with a hyperspectral camera, and a technique like the one Vivo-based is used. It captures the brain region in 128 bands, and each band consists of different information about the brain. The process of each stage of the proposed method is elaborated in the following.

The article "Investigations on Brain Tumor Classification Using Hybrid Machine Learning Algorithms" was published in 2022. Journal: J Healthc Eng.

### 3.2. Conversion of the Hyperspectral Cube to RGB Format

Our research data preprocessing is one of the common process-forming concepts for the images mapping and noise removal sections. In the HSI RGB form, images have the maximum data in every pixel and color, typically 150 to 400 dimensional vectors were analyzed and configured. The reflection of the pixel consists of each wavelength.

In this preprocessing stage, two processes were performed under the following conditions:

- Greyscale process.
- Noise removal process.

Previous research work was performed based on the greyscale process. Noise removal is acting under adaptive and Frost filters to get a better result. The adaptive filter uses an actual pixel integer concept that is replaced with an advanced pixel integer concept, and it presents better results and high performance.

### 3.3. Frost Filtering

The Frost filter exchanges the pixel of interest with the moving (nXn) kernel's total weighted values. The weighting factor decreases as one moves away from the pixel of interest. As the variance of the kernel grows, the weighting factors for the central pixels will also grow. This filter was based on the statistics of multiplication and stationary noises.

Frost filter minimizes image edges speckle content. This type of filter is a damaged symmetric regular filter used for linear data. It was determining the accurate pixel here, replacing the filter and estimation based on filter distance.

Various order speckle pictures expressed the following equation:

(1) $$\begin{array}{c} J\left(m,n\right)=a\left(m,n\right).n\left(m,n\right), \end{array}$$

where *J* (*m*, *n*) is the speckle-noise image value corruption, *a* (*m*, *n*) is the actual speckle free signal, and *n* (*m*, *n*) is the speckle noise.

### 3.4. Feature Extraction

This process is to group the regions of the brain using an optimized *k*-means clustering technique. The term optimized refers to selecting the optimal clusters value for the *k*-means clustering process. This optimization approach helps to group the different regions of the brain, along with the tumor part.

Suppose local window size is *N* × *N* means; the result is expressed as

(2) $$\begin{array}{c} s\left(i,j\right)=\;\overset{i+Nj}{\underset{K=i-Nj}{\sum }}\overset{j+N}{\underset{i=j-Nj}{\sum }}h\left(k,l\right).I\left(k,l\right), \end{array}$$

where

(3) $$\begin{array}{c} s\left(i,j\right)=\overset{i+Nj}{\underset{K=i-Nj}{\sum }}\overset{j+N}{\underset{i=j-Nj}{\sum }}h\left(k,l\right).I\left(k,l\right),\\ d_{kj}=\sqrt{{\left(i-k\right)}^{2}}+{\left(j-l\right)}^{2}, \end{array}$$

where *k* is constant.

The article "Investigations on Brain Tumor Classification Using Hybrid Machine Learning Algorithms" was published in 2022. Journal: J Healthc Eng.

### 3.5. Firefly Algorithm (FA)

Firefly algorithm is a metaheuristic algorithm for the advancement of optimization. This concept is based on the speckle action of firefly insects. Xin-She Yang introduced this algorithm in 2008. Firefly algorithm (FA) uses speckle action to impress another firefly, naturally transmitting signals to differing gender. Firefly is of a similar gender; also, all fireflies can impress another firefly. This consists of brightness for all pairs of fireflies. A brighter firefly attracts another firefly; therefore, the minimum brighter ones are replaced with the brighter ones. The algorithmic flow of the firefly is given in Table 1. The fireflies' beginnings are based on the boundary's integer concept, which is the maximum and minimum limitation statement. The maximum and minimum limitation statements of the fireflies are 1 and 5.

The formula of a pair of two fireflies is expressed as follows:

(4) $$\begin{array}{c} x_{i\;}^{t+1}=x_{1\;+\beta \text{exp}\left(-\gamma r_{ij}^{2}\right)}^{t}\left(x_{j\;-x_{i\;}^{t}}^{t}\right)+\alpha_{t\;\varepsilon_{t}}, \end{array}$$

which is optimized by

(5) $$\begin{array}{c} F\left(x\right)=\left(f1\left(x\right),f2\left(x\right),\ldots ,fi\left(x\right),\;i=1,2,3,\ldots ,m\right). \end{array}$$

### 3.6. *K*-Means Clustering

It is the function of a similar pixel integer, and it is synthesis in one part. In our research work, an unsupervised method is referred to as clustering implemented in this section. The undefined address part of a picture is addressed by presenting the *k*-means clustering function about a centric portion.

This incorporates the pixel integer term of a picture-based *k* region, where *k* is several clusters in the picture and *k* calculates the firefly optimization function. The entire process is performing under the basis iteration still in the cluster form of every pixel picture. The clustering is one of the pixel properties, and by getting the *k* value of 3, the mapping region is performed based on the threshold method.

Addressing a function of the pixel term performs a *k*-cluster state. The centric portion calculated the choosing pixel property concept and the weight of both group concepts under the clustering condition.

The code profiling was performed using the dataset created by original HS images and assuming *k* = 24, min_error = 10^−3^, and max_iter = 50.

### 3.7. Mapping the Regions

The affected region is mapped based on the neural network model, which uses a multilayer feedforward neural network. In the below discussion, the MFNN was described.

#### 3.7.1. Multilayer Feedforward Neural Network (MFNN)

Neural networks are computing systems made up of linked nodes that function similarly to neurons in the brain. Using the MFNN method, hidden patterns can be detected, correlations in raw data, cluster, and classifications can be performed, and the proposed MFNN continually learns and enhances over time. This is one of the popularised single-layer feedforward neural networks, naturally used in addressing the operation of the brain molecule. Testing the web is based on the brain's molecule and also the integer of the image. Dataset classification is based on testing and training based on the cross pleat estimation section. The neural network training is based on the training characteristics; the performance process and the results are produced based on those values.

The article "Investigations on Brain Tumor Classification Using Hybrid Machine Learning Algorithms" was published in 2022. Journal: J Healthc Eng.

In supervised learning, data labelling is an important component of data preparation. Every error or inaccuracy in this procedure might have a detrimental impact on the quality of a dataset. Furthermore, the overall performance of a predictive model might be lost, leading to errors. Taking this into account, for the ground truth in the tumor identification problem, the MFNN algorithm was applied, which labelled the data.

The multilayer feedforward neural network (MFNN) (refer to Figure 2) using the segmental feedback layer is given. The flow model is presented in the following figure. Here, it intimated the input process and the output process terms.

Multilayer feedforward neural network (MFNN) generates two classifications:

- Single multilayer feedforward neural network.
- Multiple multilayer feedforward neural network.

The single-layer MFNN is helping the performance improvement to present the result alone. Another classification is multiple MFNN is used to find the difference between real integer resultant layers through the sigmoid activation process. The sigmoidal activation function in the MFNN presents an improved output with repespect to the individual input layers. In this investigation, MFNN is utilizing the testing and training sets of the image classification configuration. Meanwhile, 80% of the samples were utilized for training and 20% for testing. Input is one of the optimal features for the FNN from the objective of the research work. The trained single-layer feedforward neural network is tested on the feature extracted image. The performance metrics evaluate the results, and they are tabulated in the experimental part.

## 4. Experimental Analysis

In this, the Matrix laboratory software is utilized to execute the proposed technique in the simulation format. The proposed method is tested on the open-access brain tumor dataset (250 samples) collected from Kaggle data collection, which is used in the parallel *k*-means clustering for better analysis and comparison [25].

The article "Investigations on Brain Tumor Classification Using Hybrid Machine Learning Algorithms" was published in 2022. Journal: J Healthc Eng.

For training and testing, the dataset is split into 80% for training and 20% for testing. The following figures are the input and output of each stage of the proposed technique. The MFNN is reconfigured based on the features extracted by our proposed method. The reconfigured network was utilized for the training and testing of the data. The output of each process of the proposed method is shown in Figures 3–6.

The RGB format of the hyperspectral image is shown in Figure 3. The noisy image (refer to Figure 4) is preprocessed with a grayscale image shown in Figure 5. This noisy signal is processed with the GLCM method.

The filtered output image is shown in Figure 6. Based on these images, the mean absolute error value and peak signal-to-noise ratio are evaluated, and they are compared with the existing method, which is depicted in Table 2.

The comparisons of the existing methods with the proposed method are made by calculating the following parameters:

  MAE: MAE is the abbreviation of mean absolute error, which tells how much percentage of the detected labels has deviated from the original labels.
  PSNR: PSNR is the abbreviation of the peak signal-to-noise ratio, which gives information about the image's quality after several processes to map the brain regions. The PSNR is increased in a hybrid firefly based on the *k*-means clustering technique by comparing the results. The results are compared with parallel *k*-means, optimized *k*-means, and SVM with *k*-means techniques. The mean absolute error is raised in the parallel *k*-means clustering technique and better in the proposed model (Table 2).

The performance evaluation was carried out in order to assess the efficiency of the proposed model. Accuracy, sensitivity, and specificity are three performance measures used in the assessment. By merging specificity and sensitivity, a single metric, quality, may be obtained. Both metrics should have a value of one. These three comparable performance measuring evaluations are also used in this study, which are as follows:

(6) $$\begin{array}{c} \text{Sensitivity}=\frac{\text{TP}}{\text{TP}+\text{FN}}\%,\\ \text{Specificity}=\frac{\text{TN}}{\text{TN}+\text{FP}}\%,\\ \text{Accuracy}=\frac{\text{TP}+\text{TN}}{\text{TP}+\text{FP}+\text{TN}+\text{FN}}\%. \end{array}$$

- TP: true positive was the total of truly identified brain tumor.
- FP: false positive was the total misclassified regions as a brain tumor.
- FN: false negative was the total from inaccurately unidentified areas.
- TN: true negative was the total of the truly identified nonbrain tumor.

The article "Investigations on Brain Tumor Classification Using Hybrid Machine Learning Algorithms" was published in 2022. Journal: J Healthc Eng.

In Table 3 and Figure 7, the comparisons of the performances analysis of the proposed model with other existing approaches were represented. Accuracy, sensitivity, and specificity are the parameters evaluated for this performance analysis. Based on the true positive and true negative values, the efficiency of the model was calculated. The proposed model is compared with *k*-NN, DNN, PSO, LSVM, and DCNN [1, 17–28]. The proposed model achieved 96.47% accuracy, which is 1.17% to 3.13% higher than other techniques, with a sensitivity of 96.32%, which is 2.06% to 5.1% better than other methods, and specificity of 98.24%, which is 0.5% to 3.6% improved compared to other techniques.

## 5. Conclusion

This research proposed an unsupervised approach for clinical treatment based on the patient's brain tumor estimation. The brain's mapping and localization are achieved using *k*-means clustering, firefly optimization, and MFNN. The proposed multilayer feedforward neural network (MFNN) addresses the brain-molecule optimization method's process and achieves minimum error and trial techniques. Hence, the proposed optimized mapping process produced improved outputs in every form, and it is suitable for mapping the molecules of the spectral medical image. The proposed model is compared with *k*-NN, DNN, PSO, LSVM, and DCNN. The proposed model achieved 96.47% accuracy, which is 1.17% to 3.13% higher than other techniques, with a sensitivity of 96.32%, which is 2.06% to 5.1% better than other methods, and specificity of 98.24%, which is 0.5% to 3.6% improved compared to other techniques. In future, to improve the performance, a hybrid deep learning method with a deep transfer learning model for the brain tumor classification process using related image datasets can be implemented. For the feature extraction process, a novel threshold-based method can be used [25–28].

## Figures and Tables

**Figure 1:** Flowchart for the mapping process.

**Figure 2:** MFNN data flow model.

**Figure 3:** RGB format of HSI image.

**Figure 4:** Noisy image.

**Figure 5:** Preprocessed greyscale image.

**Figure 6:** Postfiltered output.

**Figure 7:** Graphical view of compared performance analysis.

**Table 1:** Firefly algorithm pseudocode.

**Begin**
(1) Objective function: *f* (*x*), *x* = *x*1, *x*2,…, *Xn*;
(2) Generate an initial population of fireflies
*X*_*i*_ (*i* = 1, 2, 3).
(3) Formulate light intensity *I* so that it is associated with *f* (*x*)
(for example, for maximization problems, *I α f* (*x*) or simply *I* = *f* (*x*);)
(4) Define absorption coefficient *γ*
**While** (*t* < MaxGeneration)
**for ***i* = 1: *n* (all *n* fireflies)
**for ***j* = 1: *i* (*n* fireflies)
**if** (*i*, *j*),
Vary attractiveness with distance *r* via Exp (−𝛾, 𝑟);
move firefly *i* towards *j*;
Evaluate new solutions and update light intensity;
**end if**
**end for j**
**end for i**
Rank fireflies and find the current best;
**end while**
Postprocessing the results and visualization;
**end**

**Table 2:** Performance comparison results.

Parameters	Parallel *k*-means clustering	Optimized *k*-means clustering	SVM with *k*-means clustering	Hybrid firefly and *k*-based clustering
Mean absolute error value	75	70	68	65
Peak signal-to-noise ratio	72	75	80	85

The article "Investigations on Brain Tumor Classification Using Hybrid Machine Learning Algorithms" was published in 2022. Journal: J Healthc Eng.

**Table 3:** Comparison of performance analysis.

Classifiers	Accuracy	Sensitivity	Specificity
*K*-NN	94.93	94.26	94.55
DNN	95.30	94.85	97.70
PSO	95.11	94.71	97.01
Lagrangian SVM (LSVM)	93.34	91.22	96.69
DCNN [1]	94.50	95.10	95.86
Proposed method	96.47	96.32	98.24

## Data Availability

The datasets used and/or analyzed during the current study are available from the corresponding author on reasonable request.
